# Anti-Ulcerogenic Effect of Methanolic Extracts from *Enicosanthellum pulchrum* (King) Heusden against Ethanol-Induced Acute Gastric Lesion in Animal Models

**DOI:** 10.1371/journal.pone.0111925

**Published:** 2014-11-07

**Authors:** Noraziah Nordin, Suzy Munir Salama, Shahram Golbabapour, Maryam Hajrezaie, Pouya Hassandarvish, Behnam Kamalidehghan, Nazia Abdul Majid, Najihah Mohd Hashim, Hanita Omar, Mehran Fadaienasab, Hamed Karimian, Hairin Taha, Hapipah Mohd Ali, Mahmood Ameen Abdulla

**Affiliations:** 1 Department of Pharmacy, Faculty of Medicine, University of Malaya, Kuala Lumpur, Malaysia; 2 Department of Biomedical Sciences, Faculty of Medicine, University of Malaya, Kuala Lumpur, Malaysia; 3 Department of Chemistry, Faculty of Science, University of Malaya, Kuala Lumpur, Malaysia; 4 Institute of Biological Science, Faculty of Science, University of Malaya, Kuala Lumpur, Malaysia; 5 Center of Foundation Studies in Sciences, University of Malaya, Kuala Lumpur, Malaysia; Faculty of Pharmacy, Ain Shams University, Egypt

## Abstract

A natural source of medicine, *Enicosanthellum pulchrum* is a tropical plant which belongs to the family Annonaceae. In this study, methanol extract from the leaves and stems of this species was evaluated for its gastroprotective potential against mucosal lesions induced by ethanol in rats. Seven groups of rats were assigned, groups 1 and 2 were given Tween 20 (10% v/v) orally. Group 3 was administered omeprazole 20 mg/kg (10% Tween 20) whilst the remaining groups received the leaf and stem extracts at doses of 150 and 300 mg/kg, respectively. After an additional hour, the rats in groups 2–7 received ethanol (95% v/v; 8 mL/kg) orally while group 1 received Tween 20 (10% v/v) instead. Rats were sacrificed after 1 h and their stomachs subjected to further studies. Macroscopically and histologically, group 2 rats showed extremely severe disruption of the gastric mucosa compared to rats pre-treated with the *E. pulchrum* extracts based on the ulcer index, where remarkable protection was noticed. Meanwhile, a significant percentage of inhibition was shown with the stem extract at 62% (150 mg/kg) and 65% (300 mg/kg), whilst the percentage with the leaf extract at doses of 150 and 300 mg/kg was 63% and 75%, respectively. An increase in mucus content, nitric oxide, glutathione, prostaglandin E2, superoxide dismutase, protein and catalase, and a decrease in malondialdehyde level compared to group 2 were also obtained. Furthermore, immunohistochemical staining of groups 4–7 exhibited down-regulation of Bax and up-regulation of Hsp70 proteins. The methanol extract from the leaves and the stems showed notable gastroprotective potential against ethanol.

## Introduction

Stomach ulcer is a gastric mucosal rupture that extends via the muscularis mucosa into the submucosa or deeper [1]. For decades, this disease has been considered one of the world's most common illnesses, and it is a global problem among youths [2]. Some of the main aggressive factors that can contribute to ulcer are gastric acid, pepsin, bile salts, abnormal motility, alcohol and nonsteroidal anti-inflammation drugs (NSAID), as well as infection with *Helicobacter pylori.* However, there are several factors that can protect the stomach from ulcer formation such as mucus secretion, gastroprotective prostaglandin synthesis, bicarbonate production and normal tissue microcirculation [3], [4], [5], [6]. Reducing gastric acid production and increasing gastric mucosal protection have been the major strategies proposed for the prevention of peptic ulcer disease [7]. Ethanol-induced gastric injury is a commonly known method used in the evaluation of therapeutic potencies against gastric ulcer [8]. Ethanol causes intense lesions penetrating into the submucosa [9], enhances reactive oxygen species (ROS) formation, and depletes the mucus membrane [10], [11], [12] which renders cell death in gastric mucosal cells. Ethanol also inhibits cyclooxygenase enzyme and suppresses the output of endogenous prostaglandins [13].

Alternative and complementary medicine has gained global attention because of their widespread use in the field of medicine for treating many diseases. There are three species of the Annonaceae family which also have antiulcer activities such as *Polyalthia longifolia* cv. Pendula. [14], *Annona squamosa* L. [15] and *Annona reticulata* L. [16]. Some of these have been traditionally used to treat peptic ulcers. The protective potential of many other compounds and extracts have been evaluated according to how they enhance gastric toleration against aggressive factors such as endogenous, exogenous or infectious agents. Studies on synthetic compounds and plant extracts emphasize the importance of introducing novel herbal resources with gastroprotective healing properties.

The plant, *E. pulchrum* used in this study is a tropical plant from the Annonaceae family and it is indigenous to Malaysia [17]. Indigenous people living in remote areas of Malaysia have been using plants from the same family as this species for traditional medicine to treat various disorders such as rheumatism, cough, fever, diarrhea, malaria, asthma, edema as well as gastrointestinal disorder [17], [18]. In addition, a study by Nordin et al. (2012) has revealed that compounds of 1-(2′,3,4′-Trimethoxyphenyl) hexan-1-ol, cleistopholine and dehydroanonaine which are present in *E. pulchrum* have shown relatively strong inhibition of platelet-activating factor (PAF) with IC_50_ values of 26.6, 50.2 and 45.4 µM, respectively [19]. PAF is a potent phospholipid mediator that plays a role in the pathogenesis of inflammatory diseases of the gastrointestinal tract [20]. Therefore, *E. pulchrum* has been selected for this study in order to assess the gastroprotective potential of the methanolic extracts of leaves and stems in rats as an animal model.

## Materials and Methodology

### Omeprazole

Omeprazole as a common reference antiulcer drug [21], [22], [23] was used as a positive control in this study. This drug was obtained from the Pharmacy of the University Malaya Medical Centre (UMMC). The drug was prepared by dissolving it in Tween 20 (10% v/v) and given orally to the animals at a dose of 20 mg/kg body weight (5 mL/kg).

### Preparation of Plant Extract

*E. pulchrum* was collected from the Cameron Highlands Montane Forest (Pahang, Malaysia). Permission to enter and to collect the samples at this location was obtained from the Director of the Forestry Department of Pahang, Malaysia in October, 2011. A botanist from Universiti Kebangsaan Malaysia, the late Prof. Dr. Kamarudin Mat Salleh, identified the specimen. The voucher specimen (SM769) was deposited at the Herbarium of the Botany Department, UKM (Bangi, Malaysia). The leaves (62.0 g) and stems (65.0 g) were dried in the air and ground to mesh size 40–60. The methanolic extracts were prepared by the maceration technique. A rotary evaporator (Buchi, Switzerland) was used to evaporate the solvent from the samples. The final yield obtained from the extracts comprised 34.2% (leaves) and 7.5% (stems). The extract was then fractionated by SPE to enrich the constituent and to provide a cleaner background spectrum before being injected into the LC-MS.

### Determination of LC-MS

Analyses were performed with an Interface-Time of Flight (IT-TOF), Shimadzu using electronspray (ESI) ionization. The peaks were separated in the C-18 reversed-phase HPLC column (Waters, USA). The solvent system consisted of 10% to 100% acetonitrile (v/v) for 15 min, gradiently at a flow rate of 0.5 mL/min. The detection was accomplished using a Diode Array Detection system (DAD) Series SPD-M20A (Shimadzu). The PDA data was shown the signal at a wavelength of 254 and 350 nm.

### Animal Study

Healthy adult male *Sprague Dawley* rats (6–8 weeks age and 200–220 g weight) were used for this study. The animal house of the Faculty of Medicine, University of Malaya, Kuala Lumpur, Malaysia provided the rats. The animals were kept under standard laboratory conditions, in stainless steel cages with high floors and a wide mesh size to prevent *coprophagia.* The animals were housed under a 12 h light-dark cycle at a temperature of 25±2°C. Standard laboratory pellets and water *ad libitum* were made accessible to the animals. The animals were fasted for 24 h before the treatment to make sure their stomachs were empty. However the rats were allowed free access to water during the fasting period until 2 h before the start of the experiment. The research was approved by the University of Malaya “Animal Care and Use Committee from Laboratory Animal Science Centre, Faculty of Medicine, University of Malaya, Kuala Lumpur, Malaysia” with Ethics No. [(ISB/30/05/2012/SG (R)]. All animals were maintained according to the guidelines of the committee.

### Acute toxicity Study

An acute toxicity study was performed to determine what would be a safe dose of leaf and stem extract to give to the animals. A total of 18 adult healthy female rats were randomly selected and divided into three groups (six rats each), vehicle (10% Tween 20, 5 mL/kg), 1500 mg/kg of leaf extract and 1500 mg/kg of stem extract (5 mL/kg), respectively [24]. Before administration of the extracts, all rats were required to fast overnight. Food was withheld for a further 3 to 4 h after dosing. Observations were made after 48 hours of the extracts pretreatment to the animals by investigating any clinical and toxicological symptoms. Any mortality during the 14 days study was reported. On day 15, all animals were sacrificed by administering an over-dose of xylazine and ketamine anaesthesia. Histological and serum biochemical parameters were determined following the standard methods of OECD [25].

### Induction of Gastric Ulcer

The fasted rats were divided randomly into seven groups in which each group has six rats. Group 1, “normal control” received Tween 20 (10% v/v) orally. Group 2, “ulcer control” received Tween 20 (10% v/v) orally. Group 3, “positive control” was given 20 mg/kg omeprazole orally. The extract-tested groups (groups 4–7) received the extracts (leaves and stems) of *E. pulchrum* at doses of 150 and 300 mg/kg, respectively. An hour later, group 1 rats were given Tween 20 (10% v/v), and those in groups 2–7 were given ethanol (95% v/v) orally. After an additional hour, all rats were euthanized using an over-dose of xylazine and ketamine anesthesia and cervical dislocation technique was done to remove the stomachs. Following excision, the stomachs were placed in containers of normal saline [26].

### Macroscopic Examination of Rats' Stomachs

Stomach ulcers are characterized by long bands and bleeding lesions on the mucosal surface parallel to the vertical axis of the stomach [27]. The damage to the gastric mucosa of each rat was determined using a planimeter (10×10 mm^2^  =  ulcer area) under a dissecting microscope (1.8×). The measurement was calculated according to the number of small squares (2 mm×2 mm) covering the length and width of each lesion band as presented as total hemorrhagic area (THA), where the sum of squares ×4×1.8 =  THA (mm^2^). The percentage of total hemorrhagic reduction (THR) was calculated using the formula below, where THA_1_ and THA_2_ represent the ulcer control group and any given group, respectively. 


### Measurements of Gastric Wall Mucus

Following the modified procedure applied by Corne *et al.* [28], the gastric wall mucus of all rats was evaluated in the present study. The glandular segments of the stomachs were detached, weighed and immediately transferred to 10 mL of Alcian blue solution (0.1% w/v containing sucrose solution, 0.16 M and buffered with sodium acetate 0.5 mL, pH 5). After 2 h incubation, 10 mL sucrose (0.25 M) was added to remove the dye from the tissues using two consecutive rinses. The dye, conjugated with the gastric wall mucus, was extracted using 10 mL of 0.5 M magnesium chloride. This mixture was moderately shaken for 1 min at 30 min intervals for 2 h. The blue extract (4 mL) was then strongly shaken with 4 mL of diethyl ether. In a centrifuge adjusted to 4000 rpm, the emulsion was centrifuged for 10 min and the reading of the spectrophotometer was recorded at 580 nm to measure the quantity of Alcian blue.

### Measurement of Gastric Juice Acid Content (pH)

The gastric contents of each rat were collected and centrifuged at 4000 rpm for 10 min. The pH of the supernatant for each sample was measured using a pH meter.

### Biological Activity of Gastric Homogenate

#### Sample Preparation

The stomach tissue homogenate from each rat was prepared for determination of its biological activity. Homogenization was performed at 4°C in a teflon homogenizer (Polytron, Heidolph RZR 1, Germany) after cutting the stomach tissue into three small pieces (approximately 200 mg for each piece) and using phosphate-buffered saline (PBS) (1 g tissue/8 mL PBS). The tissue was then centrifuged at 4,500 rpm for 15 min at 4°C. The resulting supernatant was divided into aliquots and kept at −80°C to be used for the bioactivity assays.

#### Measurement of Membrane Lipid Peroxidation

Lipid peroxidation as an indicator of oxidative stress [29], [30], [31] can be estimated by the tissue level of malondialdehyde (MDA). The MDA level of the gastric tissue homogenate collected from all rats was determined using a Cayman's TBARS assay kit according to the manufacturer's protocol. Briefly, the prepared gastric supernatant which content 250 µL of RIPA buffer with protease inhibitor was used to perform the assay. A total of 100 µL of sample/positive control, 100 µL of SDS solution and 4 mL of the colour reagent were added successively into 5 mL labeled vial. The vial was then boiled for one hour. After bouling, the reaction was stop by placing in the ice bath for 10 min. The vial was centrifuging for 10 min at 1,600×g at 4°C. The supernatant was analyzed by measuring the absorbance at 532 nm. A standard curve was performed using 1,1,3,3 tetramethoxypropane.

#### Measurement of PGE_2_ Formation

For measurement of the level of prostaglandin (PGE_2_) in the stomach tissue homogenate, an aliquot of the supernatant was assayed using a Cayman's PGE_2_ EIA Kit according to the manufacturer's protocol. The purified samples containing PGE_2_ were added into 96 wells plate. Another four reagents were used to perform the assay which including EIA buffer, PGE_2_ EIA standard, PGE_2_ AChE tracer and PGE_2_ monoclonal antibody. The develop plate was carefully read to avoid the Ellman's reagent from splashing on the cover. The plate was read at a wavelength of 420 nm (Shimadzu UV-1201, Japan).

#### Measurement of Glutathione Levels

The assay was performed using Cayman's Glutathione Peroxidase assay kit. In brief, the assay was set up in the 96 wells plate. The assay buffer and co-substrate mixture should be added in non-enzymatic, positive control and samples wells. However, additional reagent such as diluted GPx was also added in the positive and samples wells. Total Glutathione content was estimated by its interaction with Cumene Hydroperoxide, and the spectrophotometer reading was taken at 340 nm.

#### Measurement of Nitric Oxide Level

Griess assay was performed to determine the nitric oxide content by measuring nitrite/nitrate concentration [32]. The supernatant was aliquoted carefully by adding vanadium trichloride 0.8% (w/v) in 1 M HCl followed by rapid addition of Griess reagent (Sigma, USA). The wavelength of the spectrophotometer was adjusted to 540 nm.

#### Measurement of Catalase Level

Measurement of catalase (CAT) level was determined using a Cayman's Catalase assay kit. In brief, the supernatant was assayed using a microtitre plate by preparing the formaldehyde standard, positive control and samples wells. Each well contains 100 µL of diluted assay buffer, 30 µL of methanol and 20 µL of standard for only formaldehyde standard well, 20 µL of catalase (positive control) and 20 µL of samples wells, respectively. Diluted hydrogen peroxide (20 µL) was added to all the wells to initiate the reactions for 20 min. The reaction was terminated by adding 30 µL of diluted potassium hydroxide for 10 min at room temperature. Finally, 10 µL of catalase potassium periodate was added and incubated for 5 min before the absorbance was monitored at 540 nm using a plate reader.

#### Measurement of SOD Activity

Superoxide Dismutase (SOD) activity was measured in the supernatant using a Cayman's assay kit according to the manufacturer's protocol. The plate set up for the assay required the SOD standard and samples wells. Briefly, 200 µL of diluted radical detector was added to all the wells, whereas 10 µL of standard and 10 µL of samples were added separately according to the particular wells. The reaction was initiated by adding 20 µL of diluted xanthine oxidase to all wells. After 20 min incubation, the plate was read by the plate reader at 440–460 nm.

#### Measurement of Protein Concentration

Following the Biuret reaction procedure described by Gornall *et al.* [33], protein concentration (mg/mL tissue) was determined in the gastric homogenate collected from all rats.

#### The Staining of Hematoxylin and Eosin

The histology of gastric tissue was evaluated by hematoxylin and eosin staining. Buffered formalin at a concentration of 10%was used to fix the specimens of gastric tissue. The specimens (5 µm thickness) were then processed in the paraffin tissue-processing machine (Leica, Germany) and finally stained with hematoxylin and eosin. Evaluation was performed under the microscope [34].

#### Immunohistochemical Staining

The protein markers Hsp70 and Bax were detected in the gastric tissues by immunohistochemistry staining according to the manufacturer's protocol (DakoCytomation, USA). A specimen 5 µm thick was cut from the stomach tissue collected from each rat and then deparaffinized and dehydrated. Glass slides treated with 3-aminopropyltrimethoxysilane (APES) were used to prepare stomach tissue sections. Following washing with the washing buffer, tissue sections were incubated for 15 min with the biotinylated primary antibody, Hsp70 (1∶500) and Bax (1∶200). Positive findings appeared as brown staining under a light microscope.

### Study of Mucosal Glycoproteins

Periodic acid-Schiff (PAS) was used in staining a 5 µm specimen of the glandular part of each stomach to assess mucus production and to evaluate changes in both acidic and basic glycoproteins [35]. The procedure was done according to the manufacturer's directions (Sigma- Aldrich, Malaysia).

### Western Blot Assay

Bradford's colorimetric method [36] was followed to determine protein concentration in the gastric homogenate prepared from each rat. The samples were then treated with Laemmili buffer (PB buffer 0.5 M, pH 6.8; glycerol, sodium dodecyl sulfate (SDS) 10%, bromophenol 0.1%, mercaptoethanol). Using sodium dodecyl sulfate polyacrylamide gel electrophoresis, equal amounts of protein concentration (200 µg/mL) from the extract (300 mg/kg) of pre-treated rats gastric tissue were separated onto 10% acrylamide gel. The proteins were then electrophoretically transferred onto a nitrocellulose membrane and incubated with specific primary antibodies, β-actin (1∶10,000), Bax (1∶1000) and Hsp70 (1∶1000). All antibodies were purchased from Santa Cruz Biotechnology, California, USA. An enhanced chemiluminescence light-detecting kit (SuperSignal West Femto Chemiluminescent Substrate, Pierce, IL, USA) was used to perform immunodetection while densiometric data were analyzed usingthe AVSoft program.

### Statistical Analysis

All results were recorded as mean ± S.E.M (n = 6). The statistical analysis of the differences between groups was performed based on Tukey HSD analysis and the one way ANOVA test (SPSS ver.20). A *p*-value less than 0.05 was recorded as being significant. All of the biological assays were done in triplicate.

## Results

### LC-MS Analysis of the Extracts

Table **1** shows the proposed compounds present in the leaf and stem extracts of *E. pulchrum*, whilst Figure **1** displays the chromatograms for each of the extracts' peaks, taking into account the fact that the classes of compounds that can be obtained from this species may present as alkaloids, acetogenins, terpenoids or steroids. Some compounds have been reported to exist in the same species and also the same genus. Therefore, compounds that are presented in both extracts of *E. pulchrum* were compared for their molecular weight of each peak which is shown in Figure **1** with compounds reported in the same species or genus. However, most of the constituents of the extracts could not be identified as they required in-depth phytochemical studies involving the isolation of pure compounds and elucidation using NMR analysis. Through observation of the HPLC chromatograms for both extracts, alkaloids were eluted at 3 to 4 min, while acetogenins at 6–8 min. Some other compounds were eluted at 9–14 minutes indicating the possibility of the presence of steroids or terpenoids, as the retention time was in the range of non-polar compounds.

**Figure 1:** Chromatographic profiles of *E. pulchrum* extracts (A–B) leaf extract constituents profile. (C–D) stem extract constituent profile.

**Table 1:** Characterization of possible compounds from each extract of *E. pulchrum* detected by LCMS-IT-TOF.

Peak no.	Compounds	*t*_R_	Exact mass	Mass ion
		(min)	(*m/z*)	(M+H/M+Na)
1A	Annonaine	3.002	2.65.3065	266.1238
1C	Cinnamic acid	4.013	148.0524	149.0464
2A, 9D	Liriodenine	3.262–3.868	275.2583	276.0653
3A, 8D	Cleistopholine	3.392	223.2268	224.0704
4A, 3C	Lysicamine	2.980–4.172	291.0895	292.0817
5A, 2C	Liridine	4.193	321.1001	322.1024
6A, 6C	Unknown	NR	NR	NR
7A, 7D	Unknown	NR	NR	NR
8A	Plagionicin C	6.210–6.515	612.8779	635.4508
9A	Plagionicin D	6.472–7.165	610.8619	635.4338
10A, 11D	Plagioneurin C	7.208–7.642	664.9524	687.4826
11A	Unknown	NR	NR	NR
12A–14A	Unknown	NR	NR	NR
12D–14D	Unknown	NR	NR	NR
15B–17B	Unknown	NR	NR	NR
15D–17D	Unknown	NR	NR	NR
18B	Plagioneurin D/E	7.1	680.9518	703.4813

NR: Not reported.

### Acute Toxicity Study

According to the results of the acute toxicity study, the animals that received doses of 1500 mg/kg of the leaf and stem extracts were still alive and had not exhibited any signs of toxicity after 14 days of study. This was confirmed by the liver and kidney histology (Figure **2**) and biochemistry results (Table **2** and **3**) where no toxicity was detected after administration of either of the two extracts of *E. pulchrum.*

**Figure 2:** Histological sections in acute toxicity test (H&E staining, 20x). Histological sections of renal (first row) and liver (second row) cells in acute toxicity test. Rats treated with 5 mL/kg vehicle (10% Tween 20) (A and D). Rats treated with 1500 mg/kg (5 mL/kg) of leaf extract (B and E). Rats treated with 1500 g/kg (5 mL/kg) of stem extract (C and F). There is no significant difference in structures of renal and liver cells between treated and control groups.

**Table 2:** Renal function test in acute toxicity study of *Enicosanthellum pulchrum* in female rats.

Dose	Sodium	Pottasium	Chloride	CO_2_	Anion gap	Urea	Creatinine
	(mmol/L)	(mmol/L)	(mmol/L)	(mmol/L)	(mmol/L)	(mmol/L)	(µmol/L)
**Vehicle**	141.88±2.45	4.812±0.14	105.37±0.54	23.17±0.63	18.06±0.51	7.85±0.33	41.03±.99
**(10% Tween 20)**							
**Leaves (1500 mg/kg)**	142.25±.68	4.48±0.19	106.62±3.63	22.29±0.70	17.26±0.68	8.08±0.81	42.11±4.84
**Stems (1500 mg/kg)**	141.59±.55	4.57±0.18	106.05±3.75	22.55±.75	17.49±0.67	8.42±0.69	42.35±4.61

Values expressed as mean ± S.E.M. There are no significant differences between groups. Significant value at p<0.05.

**Table 3:** Liver function test in acute toxicity study of *Enicosanthellum pulchrum* in female rats.

Dose	Total protein	Albumin	Globulin	TB	CB	AP	ALT	AST	GGT
	(g/L)	(g/L)	(g/L)	(µmol/L)	(µmol/L)	(IU/L)	(IU/L)	(IU/L)	(IU/L)
**Vehicle**	64.58±.27	11.21±.28	53.30±.46	2.00±.00	1.00±0.00	110.15±5.12	43.11±2.08	171.41±5.54	3.60±0.55
**(10% Tween 20)**									
**Leaves (1500 mg/kg)**	65.25±2.38	11.41±0.53	52.17±.67	2.00±0.00	1.00±0.00	98.88±4.98	40.33±.75	172.27±.15	3.42±.58
**Stems (1500 mg/kg)**	66.07±.46	10.55±.49	54.07±0.79	2.00±0.00	1.00±.00	102.32±5.67	42.65±.38	174.55±.88	3.35±.73

Values expressed as mean ± S.E.M. There are no significant differences between groups. Significant value at p<0.05.

### Macroscopic Evaluation of Gastric Lesions

The effect of both extracts on macroscopic study is shown in Figure **3**. The hemorrhagic lesions observed were confined to the glandular portions. The percentage inhibition in groups pre-treated with extracts is presented in Table **4**. The rats which received the extracts showed a significant reduction in ulcer area when compared to group 2. At high concentrations of 300 mg/kg, the % THR of the rats which received the leaf and the stem extracts was 75% and 65%, respectively. The lower concentration (150 mg/kg) showed a similar THR percentage (63% and 62% for the leaf and stem extracts, respectively).

**Figure 3:** Effect of *E. pulchrum* extracts on macroscopic appearance of the gastric mucosa in ethanol-induced gastric mucosal lesions in the groups (n = 6). (A) Normal control group shows no lesions to the gastric mucosa; (B) Ulcer control group displays severe lesions to the gastric mucosa (black arrow); (C) Omeprazole (20 mg/kg), a positive control group shows mild lesions to the gastric mucosa; (D–E) Rats receiving 150 and 300 mg/kg of stem extract show moderate lesions to the gastric mucosa, (F–G) Rats pretreated with 150 and 300 mg/kg of leaf extract show mild lesions in the gastric mucosa.

**Table 4:** Effects of *E. pulchrum* extracts on ulcer area, percentage inhibition, gastric wall mucus content and pH of gastric content.

Animal group	Pretreatment	Ulcer index	Inhibition (%)	Mucus content	Gastric pH
		(mm2)		(mg Alcian blue/g tissue)	
1	Tween 20	0	0	1.99±0.09	3.01±0.77
	(normal control)				
2	Ethanol 95%	496.5±0.11	0	1.17±0.11	1.67±0.11
	(Ulcer control)				
3	Omeprazole	115.0±6.83*	77.0*	4.62±0.09*	3.63±0.11*
	(20 mg/kg)				
4	Stem extract	190.0±4.30* #	62.0*	3.54±0.06* #	4.36±0.08*
	(150 mg/kg)				
5	Stem extract	174.83±4.49* #	65.0*	3.80±0.06* #	3.41±0.12*
	(300 mg/kg)				
6	Leaf extract	182.16±2.99* #	63.0*	3.16±0.99* #	3.12±0.74*
	(150 mg/kg)				
7	Leaf extract (300 mg/kg)	125.48±3.55*	75.0*	3.22±0.03* #	3.77±0.41*
	(300 mg/kg)				

Data were measured as mean ± standard error mean of (n = 6);

*P<0.05 compared to group 2,

# *P*<0.05 compared to group 3. All of the biological assays were done in triplicate.

### Gastric Acidity Analysis

Gastric acid content decreased significantly in groups 3–7 compared with group 2. In group 1, the acidity content showed no significant difference (*p*>0.05) compared to the group that was pre-treated with leaf and stem extracts. The stem extract at a dose of 150 mg/kg (group 4) produced a higher pH than in group 3 (Table **4**).

### Biochemical Evaluation of MDA, PGE2, Catalase and Protein Concentration

The MDA levels of the leaf extract of *E. pulchrum* (300 mg/kg) showed no significant difference (*p*>0.05) when compared with the omeprazole as positive control group. Reduction in lipid peroxidation occurred when the rats in groups 3–7 were pre-treated with extracts or omeprazole. Meanwhile, there was enhancement of PGE2, catalase and protein concentration levels in the gastric tissue homogenate from rats in groups 3–7 when compared with the ulcer control group (group 2). The stem extract at 150 mg/kg had a similar PGE2 level to omeprazole (20 mg/kg). Protein concentration levels in the gastric homogenate exhibited no significant differences (*p*>0.05) between stem and leaf extracts when they were compared (Table **5**).

**Table 5:** Observed data from biochemical analysis of MDA, PGE_2_, Catalase and protein concentration.

Animal group	Pretreatment	MDA	PGE_2_	Catalase	Protein
		(µmol/g tissue)	(ng/mg)	(nmol/min/mL)	(mg/mL)
1	Tween 20	17.43±0.41	3.52±0.12	148.22±2.89	19.13±0.52
	(normal control)				
2	Ethanol 95%	43.59±0.83	2.13±0.06	58.97±2.71	11.45±0.39
	(Ulcer control)				
3	Omeprazole (20 mg/kg)	23.26±0.49*	3.19±0.06*	146.43±2.08*	16.08±0.52*
4	Stem extract (150 mg/kg)	32.48±0.55* #	3.19±0.13*	119.77±1.08* #	14.79±0.27*
5	Stem extract (300 mg/kg)	29.07±0.38*_#_	3.23±0.06*	116.06±2.34* #	14.42±0.31* #
6	Leaf extract (150 mg/kg)	28.66±1.20* #	2.96±0.08*	108.87±2.15* #	14.34±0.41* #
7	Leaf extract (300 mg/kg)	26.37±0.96*	2.87±0.79*	138.68±2.64*	14.87±0.15*

MDA: malondialdehyde PGE2: prostaglandinE2. Data are expressed as mean ± standard error mean (n = 6);

*P<0.05 compared with group 2,

# *P*<0.05 when compared with group 3; All of the biological assays were done in triplicate.

### Antioxidant Evaluation of Stomach Homogenate

Pre-treatment with omeprazole and both extracts (150 mg/kg and 300 mg/kg) enhanced the level of antioxidant enzyme activity inthe gastric tissues. The gastric homogenates showed that the levels of GSH, NO and SOD for the pre-treated groups 3–7 were significantly increased compared to group 2 (Figure **4**). Comparison between the two extract groups for GSH level displayed a higher increment for the stem extract (300 mg/kg) compared with the leaf extract. This could have increased the level of SOD (26.57±0.87 U/mg protein) in the leaf extract compared with the stem extract (21.56±1.01 U/mg protein) when the same dose (300 mg/kg) was given to the experimental animals. Meanwhile, rats in groups 3–7 showed significant differences in NO levels (*p*<0.05) compared to rats in group 2, which were given ethanol alone.

**Figure 4:** Effects of *E. pulchrum* extracts on glutathione (GSH), superoxide dismutase (SOD) and nitric oxide (NO). Groups 1–3 represent negative control of Tween80, ethanol 95% and positive control (omeprazole, 20 mg/mL), respectively. The experimental groups from 4–7 received 150 and 300 mg/kg of stem extract and the same dosage of leaf extract. All values are expressed as standard error of mean where p<0.05 is considered significant (one between groups ANOVA with post-hoc analysis). *P<0.05 compared to group 2 and ^#^ *P*<0.05 compared to group 3. All values represent mean ± S.E.M (n = 6) and the biological assays were done in triplicate.

### Histology of Gastric Lesions

Gastric ulcer examination by H&E staining showed clear gastric mucosal damage. Some necrotic lesions also penetrated deeply into the mucosa of the ulcerated stomachs of the ulcer group. Other effects due to ethanol pre-treatment were leucocyte infiltration and extensive edema of the submucosal layer. However, groups pre-treated with *E. pulchrum* extracts exhibited remarkable protection via reduction of the ulcer area, leucocyte infiltration and submucosal edema (Figure **5**).

**Figure 5:** Histological effects of *E. pulchrum* extracts on gastric tissue (H&E staining 20×) in the groups (n = 6). Normal group shows healthy gastric mucosa (A). The ulcer control group has severe disruption to the gastric mucosa (black arrow); necrotic lesions penetrating deeply into the mucosa, extensive edema of the submucosal layer (blue arrow) and leucocyte infiltration (yellow arrow) (B). The omeprazole group shows mild damage to the surface epithelium mucosa (C). In the experimental groups, rats pre-treated with 150 and 300 mg/kg of the stem extract show mild mucosal disruption with edema and leucocyte infiltration of the submucosal layer (D–E). In the groups pretreated with 150 and 300 mg/kg of the leaf extract, rats showed a moderate mucosal disruption with edema and leucocyte infiltration in the submucosal layer (F–G).

### Mucosal Glycoprotein Evaluation

The gastric mucosa in rats pre-treated with extracts reflected a significant increase in PAS staining intensity as compared to group 2, indicating an increment in the gastric mucosal content of glycoprotein in pre-treated rats. At a dose of 300 mg/kg, the leaf extract showed greater intensity in PAS staining compared to the stem extract (Figure **6**).

**Figure 6:** Effects of *E. pulchrum* extracts on gastric tissue glycoprotein (PAS staining 20×) in the groups (n = 6). The negative control group (A); the ulcer control group (B); the omeprazole-treated group (20 mg/kg) control group (C); the experimental groups pre-treated with 150 and 300 mg/kg of stem extract (D–E) and groups pre-treated with leaf extract (F–G). Magenta color (green arrow) in the apical epithelial cells of the groups pre-treated with omeprazole (C), and extracts (D–G) shows increased intensity of mucus in gastric glands.

### Immunohistochemistry

Immunohistochemistry results for Hsp70 protein showed upregulation when pre-treated with omeprazole or the extracts (Figure **7**). On the other hand, Bax protein displayed the opposite result in those groups, which recorded significant down-regulation of the Bax protein level compared with group 2 (Figure **8**).

**Figure 7:** Effects of *E. pulchrum* extracts on the immunohistochemistry analysis of expression of Hsp70 proteins (20×) in the groups (n = 6). Normal control group (A), ulcer control group (B), omeprazole-treated group 20 mg/kg (C), rats receiving 150 and 300 mg/kg of the stem extract (D–E), rats receiving 150 and 300 mg/kg of the leaf extract (F–G). Immunohistochemistry staining of Hsp70 shows over-expression of Hsp70 protein in the experimental groups (D–G). The orange arrow points to Hsp70 protein accumulation.

**Figure 8:** Effects of *E. pulchrum* extracts on the immunohistochemistry analysis of the expression of the Bax protein in the gastric mucosa of rats in the groups (n = 6). (A) Normal control group; (B) ulcer control group; (C) positive control group, omeprazole (20 mg/kg); (D–E) Rats pre-treated with 150 and 300 mg/kg stem extract; (F–G) Rats pre-treated with 150 and 300 mg/kg leaf extract of *E. pulchrum*. Bax protein expression (red arrow) was downregulated in rats pre-treated with postive control and *E. pulchrum* extracts (magnification 20×).

### Western Blot Test

The expression levels of Bax, Hsp70 and β-actin were evaluated by western blotting analysis (Figure **9**). There were changes in each protein when treated with leaf and stem extracts. Expression of Bax was significantly higher in group 2 and lower in the extract-treated groups (*P*<0.05). The expression of Hsp70 protein was significantly increased when treated with omeprazole and extracts compared to group 2 (*P*<0.05).

**Figure 9:** Effect of leaf and stem extracts of *E. pulchrum* on Hsp70, Bax and β-actin. Groups 1 represents negative control, group 2 represents ulcer control group and group 3 represents reference standard drug. The experimental groups 4–5 received 300 mg/kg of stem and leaf extract, respectively. The statistical significance is expressed as p<0.05.

## Discussion

The study was done to find out acute toxicity in animals of leaves and stems extracts of E. pulchrum and the effectiveness these extracts to prevent the formation of gastric ulcers. Based on the observations, exhibited that these extracts have potential as antiulcer agent at the doses of 150 and 300 mg/kg. Likewise, the *E. pulchrum* plant did not show any acute toxicity in the kidney and liver of pre-treated rats that had received the leaf and stem extracts at a dose of 1500 mg/kg. A similar situation occurred with ethanol extract of *Mucuna pruriens* (L.), where no toxicity was observed in rats when a dose of 2000 mg/kg was administered [23]. Comparisons are made to the plant with previous studies to prove that natural products are non-toxic at high doses. In addition, natural products are inherently better tolerated in the body and have innate advantages for drug discovery and development [37], [38], [39], [40].

Preliminary photochemical screening of these two extracts showed the presence of alkaloids, terpenoids, phenolic compounds as well as saponins [a]. The results shown in the LC-MS chromatograms also provide an overview of the following classes of compounds. According to a study by Junaidi et al. says that active principle of antiulcer activity are flavonoids, terpenoids and tannins [41]. In addition, alkaloid compounds also reported have potent activity against gastric ulcers [42]. The previous studies by Nordin et al. [23] and Lavault et al. found several alkaloids in these plants [43]. This could explain that these classes of compounds contribute to the antiulcer activity of both *E. pulchrum* extracts. However, the alkaloids found in *E. pulchrum* had lack of documented literature on pharmacology action in experimental animal, particularly antiulcer activity. Therefore, data related to the study are able to provide guidance on the use of *E. pulchrum* as gastroprotective agents.

The use of ethanol to induce gastric ulcers predominates in antiulcer studies especially animal model studies [44], [45]. This is because ethanol easily penetrates the gastric mucosa and causes gastric ulcer [8], [46]. The damage appears on the gastric mucosa 1 h after administration of ethanol in rats [44], [45]. Gastric lesions induced by ethanol are not only associated with a decrease in gastric mucus, but also an increase in lipid peroxidation, oxidative stress inside the cells, changes in permeability and depolarization of the mitochondrial membrane, which ultimately leads to cell and membrane damage [47]. In addition, ethanol administration produces hemorrhagic lesions, infiltrated inflammatory cells, extensive submucosal edema, epithelial cell loss and mucosal friability in the stomach. These are typical symptoms of alcohol injury [48]. Therefore, application of ethanol in experimental animals has long been used as a reproducible method to induce severe lesions in the gastric mucosa [10], [49].

Omeprazole was used as the positive control drug in this study as it is widely used to protect the gastric mucosa. Several studies that have involved gastroprotective activities have used omeprazole as a positive control [50], [51], [52]. Omeprazole is a proton pump inhibitor that acts as an acid inhibitor agent in the treatment of diseases associated with gastric acid secretion [53]. In addition, omeprazole is also very effective in acid-dependent ulcer models [54]. In the ulcer model-induced by ethanol, omeprazole exhibits protection against mucosal injury at doses which do not inhibit mucus secretion [55], [56].

Based on the etiology of gastric ulcer caused by ethanol, gastric lesions could be seen on macroscopic observation, as were extensive edema and leucocyte infiltration in the histology studies for group 2 (ulcer control group). However, the production of ulcer was decreased in pre-treated rats at doses of 150 and 300 mg/kg (groups 4–7), as described in the results section above, thus proving that the gastric defense mechanism occurs in the gastric tissue of rats. Similar results were obtained by Al-Batran et al. [53] who showed that *Parkia speciosa* Hassk. extract reduced the formation of ulcers, submucosa edema and leucocyte infiltration at dosage of 100, 200 and 400 mg/kg.

There are various factors that can influence protection against gastric ulcers such as production of mucus and bicarbonate secretion [4], acid-reduction operation, and reduction in mucosal damage mediated by oxygen free radicals and associated with reactive oxygen species (ROS) including lipid peroxidation, protein oxidation, DNA damage and cell death [44], [57], [58]. Production of mucus was a major protective factor in the present study. Gastric mucus is the first layer of defense from gastric acid, and it acts as a barrier against self-digestion [59]. The results obtained in the present work showed a significant increase in mucus production in the animals pre-treated with the *E. pulchrum* extracts. Our results are further strengthened by the PAS staining experiment and evaluation of mucosal glycoproteins. The tissue sections from rats pre-treated with 150 and 300 mg/kg of the plant extracts showed intense staining, reflecting higher mucus secretion in the gastric glands. This is similar to a previous study by Abdelwahab et al. [8] of *Bauhinia thonningii* Schum. extracts where the stomach region secreted mucopolysaccharide in the gastric mucus.

High acid content is believed to cause gastric ulcer induced by ethanol [60]. The measurement of acid content can provide a good understanding of the etiology of gastric ulcer. In this study, the action of stem and leaf extracts of *E. pulchrum* was able to restore the balance of acid content in the stomachthrough the increase in pH of the gastric content as shown in the results. A similar study conducted by another group of researchers [8] displayed an increase in gastric pH in rats pre-treated with the *Bauhinia thonningii* Schum. extract in the range of ≥3.0. The increased gastric pH observed in the pre-treated rats compared to the ulcer control group (group 2) suggests the efficacy of this plant extracts in protecting the gastric tissue from ethanol injury.

Some extensive experiments have been conducted to investigate a number of mediators involved in the gastrointestinal mucosa system, which include PGE_2_ and CAT. PGE_2_ plays an essential protective role in regulating mucus secretion from the gastric mucosa [21]. The production of PGE_2_ provides a protective effect in gastric injury models [61] through the cellular integrity of the gastric mucosa. In this study, both extracts reduced gastric damage with a marked increase in the gastric mucosal PGE_2_ content in a similar manner to that observed in the study by previous researchers of the *M. pruriens* ethanol extract (Golbabapour et al. [23]. The involvement of CAT in gastric injury caused by ethanol is observed when CAT functions in the conversion of hydrogen peroxide to water [62]. Our findings showed a significant increase in both *E. pulchrum* extracts.

It was reported that Myeloperoxidase of Neutrophils catalyses the conversion of hydrogen peroxide into toxic hydrochlorus acid (HOCl) causing lipid peroxidation and cell membrane damage [63]. An increment in lipid peroxidation is associated with the formation of ROS. Malondialdehyde (MDA) is a product of lipid peroxidation and is widely used as a marker to determine the level of peroxidation lipid [64]. The studies conducted on MDA showed a significant reduction in MDA level in rats pre-treated with *E. pulchrum* extracts (groups 4–7) compared to group 2. This explains the inhibitory effect of lipid peroxidation produced by the plant extracts in our study.

Gastric ulcer also results from the involvement of reactive oxygen species (ROS) such as superoxide anions, hydrogen peroxide and hydroxyl radicals [44]. All of these radicals in turn can cause gastric oxidative stress, which plays a pivotal role in gastric hemorrhage and ulcer formation [44]. Therefore, investigation of antioxidants such as GSH, NO and SOD in leaf and stem extracts could provide a clear picture of the mechanism of action of the *E. pulchrum* extracts. In ulcer, GSH may play an important role in protecting the stomachfrom injury. In the present study, leaf and stem extracts significantly increased the GSH level, compared to group 2 (ulcer control group). Previous studies have demonstrated that the same situation occurs with the compound isolated from *Mitrella kentii* (BI.) Miq, which restores the depleted GSH level due to ethanol administration [65]. GSH could prevent tissue damage by maintaining the reactive oxygen species [66] that play an important role in inhibiting the aggressive action which can damage gastric mucosal cells [67].

Nitric oxide is a mediator that plays a crucial role in regulating the defense of the gastric mucosa by maintaining the formation of free radicals. Apart from that, NO is also involved in mucus secretion [68], inhibiting neutrophil aggregation [69] and enhancing blood flow [70]. The response of the stomach to ethanol is inhibited by increasing the production of nitric oxide, as reported in our findings. Increased levels of NO reduce the production of free radicals that ultimately result in gastric ulcer. A study by Sidahmed et al. [48] also reported the same increase in NO levels after the administration of α-mangostin from the *Cratoxylum arborescens* (Vahl) Blume species. This indicates that the extracts of *E. pulchrum* and α-mangostin share the same mechanism in preventing the formation of free radicals, which in turn secretes mucus to prevent ulcer formation.

SOD is also another antioxidant mediator of oxidative stress. Superoxide dismutase has the capability of converting superoxide to hydrogen peroxide while catalase converts hydrogen peroxide to water [61]. If free radicals such as hydrogen peroxide are produced in high quantities, the formation of gastric ulcers will occur as shown in group 2 (ulcer control group) of our study. Administration of *E. pulchrum* extracts to rats in groups 4–7 enhanced the SOD level in the present study, as well as the SOD level in the doses of ethanol leaf extract of *Jasminum Sambac* (L.), (62.5 to 500 mg/kg) [22]. The elevation of SOD level experienced in rats pretreated with the leaf and stem extracts of *E. pulchrum*, was probably due to the depletion of lipid peroxide generated from the production of ROS [67]. Therefore, these findings show that both extracts could reduce oxidative stress caused by the administration of ethanol.

The behaviour of *E. pulchrum* extracts in the gastric ulcer mechanism was also examined for expression of Hsp70 and Bax proteins through immunohistochemistry and western blot analysis. Hsp70 is a 70 kDa protein from the Hsp family that is expressed in mammalian cells [71]. Hsp70 is one of the most abundant proteins which contribute to 1±2% of total cellular protein [72]. Hsp70 plays a role in determining cell death and defending cells from oxidative stress or heat shock [73]. Our findings displayed overexpression of Hsp70 for both immunohistochemistry and western blot experiments, which was demonstrated by the pre-treated rats from groups 4–7. In contrast, the involvement of Bax protein after administration of ethanol can cause gastric injury that leads to the apoptosis of the cells [74], [75]. Apoptosis may be involved in gastric ulcer via the disturbance in the balance of apoptotic Bax proteins [76]. The leaf and stem extracts of *E. pulchrum* demonstrated downregulation of Bax protein, reducing the apoptosis in gastric cells. These findings suggest that increasing Hsp70 levels and decreasing Bax levels protect gastric cells from ethanol injury.

To sum up, the results of our study suggest that the leaf and stem extract of *E. pulchrum* can protect the rat stomach against ethanol-induced hemorrhagic superficial mucosal lesions.

## Conclusions

In conclusion, extracts from the leaves and stems of *E. pulchrum* could be potential antiulcer agents for the prevention of ulcers induced by ethanol in animal models. Both extracts are not toxic in normal cells and are not toxic when tested on animals as well. Groups pre-treated with *E. pulchrum* extracts were able to inhibit MDA and acid production, and stimulate secretion of more mucus, PGE_2_, CAT, proteins and the antioxidant enzymes which are involved in antioxidant activities such as GSH, NO and SOD. Involvement of these extracts in regulating levels of Bax and Hsp70 proteins also shows that they have potential as antiulcer agents in the discovery and development of new drugs.
